This article has been retracted.

# Clinical Practice of Cataract Special Care Standards in Nonophthalmic Wards

**DOI:** 10.1155/2022/8303606

**Published:** 2022-01-07

**Authors:** Juan Yang, Lina Yang, Yawen Chen

**Affiliations:** ^1^Ophthalmology, Shanghai Jiao Tong University Affiliated Shanghai Sixth People's Hospital, Shanghai 200235, China; ^2^Department of Nursing, Shanghai Jiao Tong University Affiliated Shanghai Sixth People's Hospital, Shanghai 200235, China

## Abstract

Cataract is a lens metabolism disease, which is caused by various factors, and leads to metamorphic lens proteins turbidity. Cataract commonly occurs in elderly patients, and majority of these patients have clinical manifestations of blurred vision and other symptoms. In this study, we explored the clinical practice and observations of cataract care criteria in nonophthalmic wards. To realize this, a total of one hundred and twenty (120) cataract patients, admitted to the East Department of Ophthalmology, Shanghai Sixth People's Hospital, particularly from April 2019-2020, were divided into the control and observation groups, where 60 cases were added to each group. The control group received routine nursing, and observation group was treated with cataract care criteria based on the control group. The complication rate, health cognition, and patient's satisfaction were compared with existing approaches. The incidence of corneal edema, anterior chamber hemorrhage, endophthalmitis, and incision infection, specifically in the observation group, was lower than that in the control group (*P* < 0.05). Likewise, the number of hospitalization days and expenses, specifically in the observation group, were lower than those in the control group (*P* < 0.05). Health knowledge and satisfaction scores of the observation group were higher than the control group (*P* < 0.05). Active service, service attitude, psychological support, caring patients, and health education dissatisfaction rate of the observation group were lower than the control group (*P* < 0.05). Finally, the standard of cataract care in nonophthalmic wards reduces the incidence of complications, improve health awareness of patients, and help to improve satisfaction of patients with nurses. Furthermore, it is worthy of promotion and application particularly in traditional hospitals.

## 1. Introduction

Cataract is a lens metabolism disease, which is caused by various factors and leads to metamorphic lens proteins turbidity. Cataract commonly occurs in elderly patients, and majority of these patients have clinical manifestations of blurred vision and other symptoms such as looking at objects and it turn dark or yellow [1]. The ocular complications might happen without prompt treatment and eventually result in blindness. The special nursing standardizations were presented under the guidance of the modern concept of holistic nursing care which integrated with the ideology of holistic nursing, targeting to continuously improving the medical care quality [2]. The unified bed management in China was first put forward by Run Shaw Hospital (RSH) affiliated to Zhejiang University Medical College, which was implemented in 1994. The standardization of medical operation, institutionalization and standardization of ward management adapting to the whole hospital operation system, and combination of general practice and specialized training of nursing staff play a significant role in the mode developing smoothly [3]. The unified bed management was proposed to solve the problem that patients cannot be admitted to hospital due to bed shortage. It includes beds of wards which were managed and allocated by the hospital, and patients can live in the vacant ward to alleviate the shortage of beds. The standardization of special disease nursing is the starting point to realize the standardization of nursing operation. The utilization rate of hospital beds has significantly increased since the implementation of the unified management system, which solved the problem of patients being hospitalized without beds. Recently, the relationship between medical care and patient, medical experience, and medical service quality are objective indicators which are likely to determine the success of China's medical reform [4]. Providing high quality standardized nursing service in different wards is a problem and needed to be solved on priority bases for improving the unified management system of beds in hospital. Therefore, in this study, we proposed a clinical practice of cataract specific nursing standards in nonophthalmic areas and tried to explore the effectiveness of the proposed model in the resolving the aforementioned issue such as provision of high-quality nursing service to the admitted patients in the hospital. Main contributions of this manuscript are highlighted.

1. Development of clinical practice which is specifically designed for cataract nursing standard adopted in traditional hospitals
2. To enhance nursing service standard which is provided to the admitted patients in various hospitals
3. Design of sophisticated procedures to resolve and improve nursing service structure in the traditional hospital in general and smart technology-based hospital in particular

The rest of the manuscript is organized according to the following procedure.

In Section 2, datasets and proposed methodology, used to enhance nursing service in hospital, is presented along with clinical data.

## 2. Proposed Data and Methods

In this section, a detail description of the dataset and proposed methodology is provided. Initially, clinical data are discussed in detail, followed by the proposed model, which is present to resolve the low-quality nursing issue associated with the admitted patients in the hospitals.

### 2.1. Clinical Data

A total of 120 cataract patients were selected in the East Department of Ophthalmology of Shanghai Sixth People's Hospital specifically from April 2019 to 2020. Cataract patients were assigned to the ward according to bed management regulations of the underlined hospital and designed by single-blind experimental. Patients in general surgery and orthopedic wards were the experimental group, and patients in the neurosurgery and urology wards were the control group with 60 cases in each group.

34 males and 26 females with an average of (61.24 ± 4.60) years were included in the control group. In the experimental group, 33 were males and 27 were females with an average of 67.78 ± 4.30 years. There was no significant difference in basic information between 2 groups (*P* > 0.05).

### 2.2. Inclusion and Exclusion Criteria

The inclusion criteria were as follows:

1. Patients in accordance with the classification and grading standards of the World Health Organization for lens opacity
2. All patients were confirmed by visual acuity examination, electroretinogram, and fundus examination
3. Patients hospitalized for the first time with junior high school education or above

The exclusion criteria were as follows:

1. Patients with severe ophthalmic diseases
2. Those who were combined with cognitive impairment or unable to fill in the questionnaire
3. Patients who need referral, hospital transfer, or discharge due to some reasons are removed from the group or automatically dropped from the group

### 2.3. Proposed Methodology

Patients in the control group were provided with routine ophthalmic nursing care. The dangers of the disease were illustrated to not only the patients but also their families. Explain the upcoming treatment to patients so as to obtain the support and cooperation of the patients as much as possible. Patients in the experimental group received cataract ZhuanBing nursing care besides routine ophthalmic nursing care. The nursing group for cataract patients was established on the basis of Ophthalmology Clinical Nursing Manual published by Scientific and Technical Literature Press in 2008. The members of the group included medical and nursing experts, head nurses, and specialist nurses. Moreover, the cataract ZhuanBing nursing standards were formulated upon the patients' disease conditions. Taking the time period as the vertical axis, the whole hospitalization process of patients was divided into five stages: admission, preoperative, intraoperative, postoperative, and discharge. The work content and indicators that need to be completed by nurses at each stage are refined and quantified. In addition, the scoring table is made to objectively evaluate the overall nursing level of patients from admission to discharge for the specialized nursing is more standardized, scientific, and specific. Each member has a clear division of labor:

- The environment in wards and hospitals were depicted to patients when admissions. Given patients still do not understand much about the disease, nursing knowledge correlated with the disease is consistently preached to improve patients' cognition and cooperation. Make more communication with patients and answer the questions raised by patients patiently in order get the relationship between patients and nursing staff closer.
- Patient's psychological state of preoperative was assessed, and timely eliminate or alleviate the negative emotions of the patient through psychological counseling when patient has been found to have negative emotions. Antibiotic eye drops were dropped for three days prior to surgery, and the eyelashes were cut one day before the operation. The lacrimal duct was irrigated with normal saline to observe whether the patient had purulent secretions in the lacrimal duct. Then, the antibiotic eye drops were dropped 4–6 times, and 10 ml normal saline was used to irrigate the lacrimal duct twice a day.
- During the operation, five patients who had irrigated the lacrimal duct and conjunctival sac walk into the operating room lying on the operating table with a proper position under the assistance of nurses. After the surgery, patient came out of the operating room safely and was evaluated psychologically again. Additionally, patients were informed the operation succeeded and provided psychological guidance to comfort patients. The relevant precautions after surgery were explained to patients such as avoiding strong light exposure and inhibiting rub the eyes and lowering the head to pick up objects. The local conditions of the patient's eyes in the operation area after surgery were observed, and notice the doctor immediately when abnormality occurs, and then take corresponding treatment measures. After the operation, patients were instructed to follow doctor's advice to take medicine and directed the patient and their families to conduct eye drops correctly.
- Most patients are discharged from hospital within three days after postoperative guidance and complete the discharging formalities assisted by nurses. Information for patients return home involves good hand hygiene, increase exercise appropriately, and do not wipe eyes with hands or handkerchiefs and lower head to take objectives or wash hair to keep the eyes in no contact with water. More importantly, patients should avoid having too much spicy food. Remind the time for recheck of the patients, and return visit cards stating the time, considerations, and relevant nursing care were issued to patients. The patient's mental state, appetite, and sleep were inquired regularly following call back.

### 2.4. Observation Indicators

(1) Complication rate: the incidence of corneal edema, anterior chamber hemorrhage, endophthalmitis, and incision infection were recorded
(2) Patients' satisfaction with nurses: based on the survey of inpatients' satisfaction with nurses in grade hospitals of nursing, quality stipulated in hospital evaluation standards of the Ministry of Health combined with the actual situation of our hospital and patients' requirements for nursing work and survey of inpatients' satisfaction with nurses were formulated. The content includes evaluation of nurses' satisfaction from the aspects of active service, service attitude, psychological support, caring for patients, and health education, and through qualitative:
  - Satisfied
  - Quite satisfied
  - General dissatisfied
In the investigation of various indicators, the total score of the questionnaire is 100, the score ≥90 is satisfied, and the number of satisfied cases is counted.
(3) Nurse skills compare science and technology literature publishing house, 2008, “ophthalmic clinical care manual” as the main basis, with the actual situation of our hospital ophthalmology and cataract patients to nursing work requirements, formulated the dispense operation scale, operation scale shear eyelash, flush the conjunctival sac operation scale, and operating points such as 80 and 20 points for theory. The nurses in both experimental and control groups were assessed, and the average score was counted.

### 2.5. Statistical Analysis

In the proposed model, SPSS14.0 software was used for the statistical analysis. The counting data were represented by *N* (%), and measurement data were represented by the *t*-test. *P* < 0.05 was statistically significant.

## 3. Experimental and Simulation Results

In this section, a comprehensive and thorough analysis of various experimental or simulation results has been presented. Additionally, comparative analysis is presented in separate subsection (Table 1).

### 3.1. Comparison of Complication Rate between Two Groups

Table 1 provides the details of the comparison of complication rates between two groups.

### 3.2. Comparison of Nursing Service Satisfaction between Two Groups

The results of active service, service attitude, psychological support, caring for patients, and dissatisfaction rate of health education in the experimental group were higher than those in the control group (*P* < 0.05) (Table 2).

### 3.3. Comparison of Nurses' Operational Skills between Two Groups

The experimental group achieved higher results in dispensing eye medicine, eyelash clipping, and rinsing conjunctival sac than the control group (*P* < 0.05) (Table 3).

## 4. Discussion

Cataract is a lens metabolism disorder which is induced by various factors such as aging, genetic, local nutritional disorders, immunity and metabolic abnormalities, and radiation. Serious may present lens protein degeneration turbid. In a cataract, light is blocked from reaching the retina by cloudy lens, and thereby, patient cannot see clearly. Currently, cataract is mainly treated by surgical treatment. However, preoperative and postoperative nursing has a great impact on ensuring surgical efficacy [5]. In this study, nursing standard of cataract specific disease was applied to the nursing of ophthalmic patients in nonophthalmic areas. Cataract special nursing is a modern holistic nursing model, which makes a holistic nursing plan from various aspects.

In recent years, cataract specialist nursing has been applied in patients with a variety of diseases, and the effect is ideal. The incidence of corneal edema, anterior chamber bleeding, endophthalmitis, and infection of incision in the experimental group is lower than the control group, suggesting the cataract ZhuanBing standards of care in the ophthalmology ward nursing process through strengthen health education to patients and family members of the propaganda may effectively ensure patients' rights of knowing the fact of treatment and improve the patients' cognition [6–8].

Clinical studies indicate that the negative emotions of patients were eliminated or relieved by cataract-specific nursing, and the self-management ability of patients was promoted obviously and then to ensure the therapeutic effect of patients [9, 10]. In this study, the satisfaction score of the experimental group was higher than that of the control group (*P* < 0.05), indicating that the treatment effect and patient satisfaction were improved significantly after the application of cataract specific nursing standards in nonophthalmic wards. The excellent nursing services and humanized nursing services for patients were provided based on cataract specialist nursing standards and enhanced the quality of care [11, 12]. After surgery, the active nursing service, service attitude, health education, psychological support, and patient nursing satisfaction in the experimental group were lower than those in the control group (P <0.5). In the nursing process of implementing the cataract referral nursing standard in the ophthalmic ward, the medical staff took the initiative to serve the patients, answer the patients' questions, help the patients solve various practical problems, and improve the image of the medical staff. The results of active services, service attitude, health education, psychological support, and patients care satisfaction rate in the experimental group were apparently higher than in the control group, demonstrating that medical staff actively and patiently answer all kinds of doubts for patients and assist patients solve various practical problems in the process of implementing the cataract ZhuanBing standards of care in ophthalmology wards. Importantly, health promotion for patients not only strengthens communication between each other but also meets patients' requirements, which helps to reduce medical disputes, improve patients' satisfaction with medical staff and their own image, and increase social benefits [13, 14].

Finally, nursing standard of cataract specific diseases can reduce incidence of complications in nonophthalmic ward and help to improve the score of ophthalmic operation skills of nurses in nonophthalmic wards. The improvement of nurses' knowledge of ophthalmological operations in nonophthalmic wards is benefit to improve patients' satisfaction with nurses, which is worth promoting.

## 5. Conclusion and Future Work

In this study, we have explored the clinical practice and observations of cataract care criteria in nonophthalmic wards. To realize this, a total of one hundred and twenty (120) cataract patients, admitted to the Department of Ophthalmology, Shanghai Eastern People's Hospital, particularly from April 2019 to 2020, were divided into the control and observation groups where 60 cases were added to each group. The control group received routine nursing, and the observation group was treated with cataract care criteria based on the control group. The complication rate, health cognition, and patient's satisfaction were compared with existing approaches. The incidence of corneal edema, anterior chamber hemorrhage, endophthalmitis, and incision infection, specifically in the observation group, was lower than that in the control group (*P* < 0.05). Likewise, the number of hospitalization days and expenses, specifically in the observation group, were lower than those in the control group (*P* < 0.05). Health knowledge and satisfaction scores of the observation group were higher than the control group (*P* < 0.05). Active service, service attitude, psychological support, caring patients, and health education dissatisfaction rate of the observation group were lower than the control group (*P* < 0.05). Finally, the standard of cataract care in nonophthalmic wards reduces the incidence of complications, improve health awareness of patients, and help to improve satisfaction of patients with nurses. Furthermore, it is worthy of promotion and application particularly in traditional hospitals.

In future, we will investigate how the proposed model is useful in improving the overall service structure of a traditional hospital.

## Figures and Tables

**Table 1:** Comparison of complication rates between two groups.

Group	Cases	Corneal edema	Anterior chamber bleeding	Endophthalmitis	Infection
Experimental group	60	1 (1.67)	0 (0.00)	1 (1.67)	1 (1.67)
Control group	60	3 (5.00)	4 (6.67)	4 (6.67)	3 (5.00)
*X* ^2^		5.691	4.396	9.124	4.311
*P*		0.034	0.029	0.014	0.037

**Table 2:** Comparison of nursing service satisfaction between two groups (*N* (%)).

Group	Satisfaction	Active service	Service attitude	Support	Patient care	Health education
Experimental group	60	60	59	58	59	58
Control group	60	51	50	52	52	53
*x* ^2^		5.331	6.390	7.410	4.897	6.534
*P*		0.023	0.012	0.015	0.020	0.023

**Table 3:** Comparison of nurses' operational skills between two groups $\left(\bar{x}\pm s\right)$.

Group	Cases	Eye medicine operation score	Eyelash cutting operation score	Irrigating conjunctival sac operation score
Experimental group	28	86.1 ± 5.01	90.88 ± 3.68	91.85 ± 3.29
Control group	29	91.22 ± 3.26	93.72 ± 3.17	93.94 ± 3.11
*F*		15.14	9.79	9.41
*P*		*P* < 0.05	*P* < 0.05	*P* < 0.05

## Data Availability

The datasets used and analyzed during this study are available from the corresponding author upon request.
